The article "Effects and Safety of Traditional Chinese Medicine for Hidden Blood Loss after Total Hip Arthroplasty—A Systematic Review and Meta-Analysis" was published in 2022. Journal: Evid Based Complement Alternat Med.

# Effects and Safety of Traditional Chinese Medicine for Hidden Blood Loss after Total Hip Arthroplasty—A Systematic Review and Meta-Analysis

**DOI:** 10.1155/2022/6937295

**Published:** 2022-08-05

**Authors:** Ze Yang, Xiang Wang, Zheyun Xu, Qike Xu, Yongliang Xia, Weifeng Ji

**Affiliations:** ^1^The First Clinical Medical College, Zhejiang Traditional Chinese Medical University, Hangzhou 310053, China; ^2^Department of Orthopedics, Tongde Hospital of Zhejiang Province, Hangzhou 310012, China; ^3^The Fourth Clinical Medical College, Zhejiang Traditional Chinese Medical University, Hangzhou 310053, China; ^4^Department of Traditional Chinese Medicine, Hangzhou Zelin Health Management Co. Ltd., Neighborhood Good Doctor No. 6 Street Clinic, Hangzhou 310000, Zhejiang, China; ^5^Department of Internal Traditional Chinese Medicine, The First Affiliated Hospital of Zhejiang Chinese Medical University, Hangzhou 310006, Zhejiang, China; ^6^Department of Orthopedics, The First Affiliated Hospital of Zhejiang Chinese Medical University, Hangzhou 310006, Zhejiang, China

## Abstract

**Background:**

Hidden blood loss (HBL) after total hip arthroplasty (THA) would lead to many undesirable consequences. Traditional Chinese medicine (TCM) is now increasingly used for hidden blood loss. We performed this systematic review and meta-analysis to summarize the effect and safety of TCM treatment of HBL after THA.

**Methods:**

We searched PubMed, Embase, Cochrane Library, CNKI, VIP, WanFang, and CBM for the updated articles published from the inception of each database to May, 2022, among which results such as abstracts, comments, letters, reviews, and case reports were excluded. The efficacy and safety of TCM treatment of HBL after THA were synthesized and discussed by the outcomes of total blood loss (TBL), hidden blood loss (HBL), hemoglobin (Hb), and hematocrit (HCT), and the incidence of adverse reactions.

**Results:**

A total of 12 articles and 881 patients were included. There were 441 cases in the intervention group and 440 cases in the control group. Compared with the control group, the intervention group had more advantages in TBL (MD = −251.68, 95% CI = [−378.36, −125]; *Z* = 3.89, *P* < 0.00001), HBL (MD = −159.64, 95% CI = [−252.56, −66.71]; *Z* = 3.37, *P*=0.0008), Hb (MD = 11.39, 95% CI = [7.35, 15.43]; *Z* = 5.53, *P* < 0.00001), and HCT (MD = 2.87, 95% CI = [0.97, 4.78]; *Z* = 2.95, *P*=0.003), and had less incidence of adverse reactions (OR = −0.20, 95% CI = [−0.35, −0.05]; *Z* = 2.64, *P*=0.008).

**Conclusion:**

TCM has advantages in the efficacy and safety of treating hidden blood loss after THA. The strength of the evidence of the research results is limited by the quality of the included literature, and more high-quality RCTs are needed to confirm.

## 1. Introduction

Total hip arthroplasty (THA) is the most commonly used and effective treatment for femoral neck fractures, hip arthritis, developmental dysplasia of the hip, and ischemic necrosis of the femoral head [1]. THA is always accompanied by blood loss, including intraoperative blood loss and postoperative blood loss, as well as some hidden blood loss (HBL) [2]. Sehat et al. [3]reported that HBL after THA was 49% of the total blood loss (TBL), since which surgeons learned that HBL plays an important role in surgery [4, 5].

HBL refers to the accumulation of blood in the joint cavity, or extravasation into the interstitial space, and the loss of hemoglobin (Hb) in the body caused by factors such as traumatic stress and other factors that induce hemolysis [6], of which the clinical manifestations are swelling, ecchymosis, and a significant decrease in Hb [7, 8]. It is one of the main causes of postoperative anemia in patients [9], which can affect the functional recovery and quality of life of the patient after surgery, and even increase the risk of infection and death, or extend the length of hospital stay [10]. Clinically, intraoperative and postoperative intravenous tranexamic acid (TXA) and other hemostatic drugs are often used to reduce HBL [5]. However, it has been reported that sometimes blood loss is not effectively controlled by these methods and with several complications [11]. There are increasing research studies reported using traditional Chinese medicine (TCM) theory to treat patients who suffer from blood loss according to symptoms and signs [12–14]. The main objective of this study was to evaluate the clinical efficacy and safety of TCM in treating HBL after THA.

## 2. Materials and Methods

### 2.1. Data Source

We searched PubMed, Embase, Cochrane Library, CNKI, VIP, WanFang, and CBM for the updated articles published from the inception of each database to May 1st, 2022. When duplicate publications were identified, we chose the most complete and recent trial. Two investigators (Z.Y. and X.W.) independently retrieved the related studies in the database and excluded duplicate publications. The combined text and medical subject heading (MeSH) terms were cross-searched using MeSH and free words as follows: (((Hidden blood loss[Title/Abstract]) AND ((((Hip Prosthesis Implantation[Title/Abstract]) OR (Hip Replacement, Total[Title/Abstract])) OR (Total Hip Arthroplasty[Title/Abstract])) OR (“Arthroplasty, Replacement, Hip”[Mesh]))) AND ((((Decoction[Title/Abstract]) OR (Tang[Title/Abstract])) OR (Fang[Title/Abstract])) OR ((“Medicine, Chinese Traditional”[Mesh]) OR ((Chung I Hsueh[Title/Abstract]) OR (Traditional Chinese Medicine[Title/Abstract]))))) AND ((randomized controlled trial [Publication Type] OR randomized [Title/Abstract] OR placebo [Title/Abstract]))

### 2.2. Inclusion and Exclusion Criteria

Inclusion criteria are as follows: (1) Type of Study: the study must be a randomized controlled trial (RCT); (2) Participants: patients receiving THA; (3) Intervention measures: the intervention group must be treated with TCM (decoction, capsule, ointment) or combined with western medicine, and the control group is treated only with western medicine; and (4) Outcomes: TBL, HBL, Hb, hematocrit (HCT), and incidence of adverse reactions.

Exclusion criteria are as follows: (1) studies are not RCTs; (2) patients not receiving THA; (3) incomplete or unidentified data; (4) duplicate publications; and (5) abstracts, reviews, case reports, and letters.

### 2.3. Study Selection and Data Extraction

Two independent researchers (Z.Y. and X.W.) read the title, abstract, and full text, screened the literature according to the inclusion and exclusion criteria, and cross-checked the results. If there is a disagreement, the third researcher (Y.L.X.) will be consulted. Extract data from the included literature, including first author, sample size of the study, gender, mean age or age range, intervention protocol, duration time, and outcomes.

### 2.4. Quality Assessment

The quality of the included studies was assessed by The Cochrane Risk Bias Tool in the Cochrane Handbook for Systematic Reviews of Interventions. The following messages were evaluated: random sequence generation, allocation concealment, blinding of participants and personnel, blinding of outcome assessments, incomplete outcome data, selective reporting, and other biases.

### 2.5. Statistical Analysis

RevMan5.4 and Stata15.0 software was used for statistical analysis. The included studies are tested for homogeneity. Pooled odds ratios (OR) and 95% confidence intervals (95% CI) were calculated to report dichotomous data, and mean differences (MD) with 95% CI were used to report continuous data. Statistical heterogeneity was considered present when *P* < 0.1 or I^2^ > 50%. When high heterogeneity existed, a random-effects model was used for meta-analysis. Sensitivity analysis was also used to analyze the source of heterogeneity. Publication bias was evaluated visually by funnel plots and considered significant when *P* < 0.05 in either Begg's test or Egger's test when the inclusion was more than 10 articles.

## 3. Results

### 3.1. Search Results

Our initial search yielded 85 articles in total, 32 of which were removed for duplication. After screening titles and abstracts, a further 17 items were taken away. 36 articles were reviewed, among which 12 were included in this meta-analysis [15–26]. No further study was identified by manual search. The flow diagram of study selection was shown in Figure 1.

### 3.2. Study Characteristic

12 studies with a total of 881 subjects were included in the meta-analysis. The outcomes of the studies are shown as follows: TBL, HBL, Hb, HCT, and incidence of adverse reactions. The main characteristics of the 12 articles were summarized in Table 1.

### 3.3. Quality of the Evidence

The results of the risk of bias assessment for all included studies are summarized in Figure 2. Randomization was used in all articles, six studies [15, 16, 19, 22, 25, 26] used the means of random number table, two studies [17, 20] grouped according to the odd-even number of admission case numbers, one study [23] used random and double-blind methods, one study [21] using the envelope method, were considered to have a low risk of bias in the random sequence generation domain. One study [18] grouped according to the treatment method was considered to have a high risk of bias in the random sequence generation domain and blinding of participants and personnel. One study [24] did not mention random methods were considered to have an unclear risk of bias. Two studies [23, 25] mentioned blinding of participation and outcome assessment were considered as low risk, while others were not mentioned, thus they were considered to have an unclear risk of bias. One study [21] had lost to follow-up cases and was considered high risk, and the rest of the studies were complete with data and considered as low risk. The selective reporting and other bias in the included articles resulted in an unclear risk of bias.

### 3.4. Outcome Measures

#### 3.4.1. TBL

9 studies [15–18, 21–25] involving 550 participants reported the outcome of TBL. Heterogeneity test analysis suggested that there was heterogeneity (*P* < 0.00001, I^2^ = 98%). The sensitivity analysis was carried out one by one, and it was found that there was no significant change, thus the random effects model was used. The meta-analysis demonstrated there was a significant difference between the two groups (MD = -251.68, 95% CI = [−378.36, −125]; *Z* = 3.89, *P* < 0.00001) (Figure 3).

#### 3.4.2. HBL

12 studies [15–26] involving 881 participants reported the outcome of TBL. Heterogeneity test analysis suggested that there was heterogeneity (*P* < 0.00001, I^2^ = 99%). The random effects model was used. The HBL in the intervention group was less than that in the control group (MD = -159.64, 95% CI = [−252.56, −66.71]; *Z* = 3.37, *P*=0.0008) (Figure 4(a)).

Subgroup analysis showed that TCM for tonifying qi and blood and TCM for activating blood stasis both have a significant difference in HBL (Figure 4(b)), which was consistent with the results reported in every study. However, both groups have high heterogeneity, which may be due to the differences in the duration and time of the research.

#### 3.4.3. Hb

9 studies [15, 16, 18–21, 23–25] involving 661 participants reported the outcome of Hb. Heterogeneity test analysis suggested that there was heterogeneity (*P* < 0.00001, I^2^ = 88%). The sensitivity analysis was carried out one by one, and it was found that there was no significant change, thus the random effects model was used as well. The meta-analysis demonstrated there was a significant difference between the two groups (MD = 11.39, 95% CI = [7.35, 15.43]; *Z* = 5.53, *P* < 0.00001) (Figure 5).

#### 3.4.4. HCT

4 studies [15, 18, 21, 22] compared HCT after TCM treatment with the control group, involving 270 participants. Heterogeneity test analysis suggested that there was heterogeneity (*P*=0.04, I^2^ = 64%). The sensitivity analysis was carried out one by one, and it was found that there was no significant change, thus the random effects model was used. The HCT in the intervention group was more than that in the control group (MD = 2.50, 95% CI = [1.28, 3.71]; *Z* = 4.03, *P* < 0.00001) (Figure 6).

#### 3.4.5. Incidence of Adverse Reactions

One study [24] involving 90 participants reported the incidence of adverse reactions to TCM. The intervention group was safer than the control group (OR = −0.20, 95% CI = [−0.35, −0.05]; *Z* = 2.64, *P*=0.008) (Figure 7).

### 3.5. Publication Bias

The publication bias of outcomes was evaluated using funnel plots based on the HBL of 12 studies. The funnel plot (Figure 8), which was asymmetrically distributed on both sides, and the Egger's test (*P*=0.001) of the HBL suggested that there was potential publication bias in the included studies.

## 4. Discussion

THA is recognized as one of the most effective surgical methods for the treatment of end-stage hip joint disease [27]. There are different degrees of hidden blood loss after surgery [28]. HBL refers to the effective circulation of hemoglobin and red blood cells entering the interstitial space after the operation, resulting in swelling of the affected limb which is not directly lost to the outside world. The hazards of hidden blood loss include postoperative anemia and complications such as slow wound healing, poor functional recovery, and increased risk of infection caused by anemia [29, 30]; increased risk of deep vein thrombosis in the lower extremities; increased probability of cardiovascular and cerebrovascular accidents; and subcutaneous ecchymosis [31]. Hidden blood loss falls into the category of “blood syndrome” in clinical Chinese medicine and can be traced back to “The Yellow Emperor's Classic of Internal Medicine.” It said: “injury of YANG-collateral leading to outwards bleeding…yin collateral impairment causing hematocheiza”.

The “yin collateral impairment” and “hematocheiza” described here are actually the same as the hidden blood loss described today. Blood circulating out of the vessels that cause swelling of the affected limb after the operation is called blood stasis. In this case, TCM thinks the bleeding cannot be stopped blindly but should remove blood stasis and stop it. In “A Treatise on Blood Troubles,” a famous classic TCM book on blood syndrome proposed four methods of treating blood syndrome: hemostasis, removing blood stasis, tranquilizing blood, and invigorating deficiency, which have been used by future generations to this day. Therefore, to treat blood syndrome, it is necessary to distinguish the cause of it. It could be caused by the stagnation of qi that blocks the normal flow of blood in the vessels, the deficiency of qi to promote blood circulation, or blood deficiency that leads to the inability to fill the vessels, so the flow rate slows down. Different etiologies and syndromes have different methods of differentiation and treatment.

This study systematically reviewed the clinical efficacy and safety of TCM in the treatment of HBL after THA. A total of 12 articles were included for the meta-analysis. The included studies used Bazhen Decoction, Tanshinone Capsules, Sanqi Zhixue Decoction, Taohong Siwu Decoction, Yiqi Huoxue ointment, Fuyuan Decoction, Yunnan Baiyao, Shiquan Dabu Decoction, and Chuanxi San to treat HBL. The prescriptions used are regulating qi and activating blood stasis to stop bleeding, tonifying qi and blood to stop bleeding, and all treatments were from the cause of blood syndrome. Therefore, the subgroup analysis showed that whether taking TCM for tonifying qi and blood or activating blood stasis, the HBL in the intervention group was smaller than the control group. The results of the meta-analysis showed that TCM has more advantages in TBL, HBL, Hb, HCT, and the incidence of adverse reactions after THA, and the difference is statistically significant.

Our review has several limitations. First, the sample size of this meta-analysis was relatively small. As a result, the unknown risk of bias caused by incomplete data could constrain our results. Second, due to the large heterogeneity of the included studies, only a random effect model can be adopted, which will have a certain impact on the results. Third, the intervention protocol varied significantly in the duration of treatment time, ranging from 7 to 30 days, and the type of intervention TCM varied from each other (capsule, decoction, ointment). At the same time, the control group received different interventions as well, which may be the reason for the high heterogeneity.

Despite these limitations, this meta-analysis provides information on the association between TCM and HBL after THA.

## 5. Conclusion

In conclusion, this article shows that TCM is more effective and safer than Western medicine in treating HBL after THA. Therefore, in the clinical treatment of HBL after THA, TCM should be added to the conventional treatment to improve the clinical efficacy. However, due to the small number of included studies and their low quality, our conclusions remain to be confirmed by further high-quality RCTs.

## Figures and Tables

**Figure 1:** PRISMA flow diagram of the study selection process.

**Figure 2:** Risk of bias graph.

**Figure 3:** Forest plots for TCM on TBL.

**Figure 4:** (a) Forest plots for TCM on HBL. (b) Forest plots and subgroup analysis of duration time for TCM on HBL.

**Figure 5:** Forest plots for TCM on Hb.

**Figure 6:** Forest plots for TCM on HCT.

**Figure 7:** Forest plots for incidence of adverse reactions.

**Figure 8:** Funnel plots of the HBL.

**Table 1:** Characteristics of the 12 studies included in the meta-analysis.

Study	Sample size (IG/CG)	Gender (Men/Women)		Mean age or age range		Intervention Protocol		Duration time	Outcomes
		IG	CG	IG	CG	IG	CG		
Cai2020	36/36	-	-	69.03 ± 5.64	70.39 ± 5.51	Sanqi zhixue Decoction combined TXA	TXA	7 days	①②③④
Ji2019	15/15	6/9	6/9	69.73 ± 0.79	70.87 ± 1.65	Bazhen Decoction combined TXA	TXA	14 days	①②③
Ke2017	30/30	11/19	14/16	71.1 ± 8.3	66.8 ± 10.1	Taohong Siwu Decoction combined TXA	TXA	7 days	①②
Li2022	37/34	26/11	24/10	77.2 ± 7.7	79.6 ± 9.3	Yiqi Huoxue ointment combined TXA	TXA	7 days	①②③④
Ma2018	53/54	24/29	26/28	71.99 ± 7.29	72.03 ± 7.31	Bazhen Decoction combined TXA	TXA	14 days	②③
Miao2017	62/62	38/24	41/21	75.67 ± 8.32	73.72 ± 7.83	Fuyuan Decoction	TXA	7 days	②③
Qiu2018	30/30	20/10	22/8	64.25 ± 2.56	64.23 ± 2.54	Yunnan Baiyao combined TXA	TXA	7 days	①②④
Qiu2019	33/34	19/16	18/17	69.13 ± 3.26	68.62 ± 3.18	Bazhen decoction combined TXA	TXA	14 days	①②③④
Sheng2017	20/20	6/14	7/13	68.7 ± 5.33	70.7 ± 4.68	Addition of Shiquan Dabu Decoction	Anti-infection and anticoagulation	14 days	①②③
Wang2015	45/45	22/23	21/24	66.0 ± 6.7	66.2 ± 6.5	Tanshinone Capsules	Low molecular weight heparin	7 days	①②③⑤
Xiao2020	30/30	9/21	8/22	65.6 ± 4.8	66.2 ± 5.2	Sanqi zhixue Decoction	No hemostatic drugs	14 days	①②③
Zhou2019	50/50	20/30	22/28	52–70	50–70	Chuanxi San combined TXA	TXA	30 days	②

CG: control group; IG: intervention group “-”: not mentioned ① TBL, ② HBL, ③ Hb, ④ HCT, ⑤ Incidence of Adverse Reactions.
